# A Power System Harmonic Problem Based on the BP Neural Network Learning Algorithm

**DOI:** 10.1155/2022/7247881

**Published:** 2022-08-16

**Authors:** Qianqian Yue, Rui Hu, Xiaoling Zhang

**Affiliations:** ^1^Anhui Sanlian College of Electrical and Electronic Engineering, Anhui, Hefei 230601, China; ^2^Wanda Tire, Anhui, Hefei 230601, China; ^3^Anhui Sanlian College of Robotics Engineering, Anhui, Hefei 230601, China

## Abstract

At present, due to the large-scale use of different kinds of power electronic devices in the power system, the problem of harmonic pollution in the power grid is becoming more and more serious, which will lead to a serious decline in the production, transmission, and utilization rate of electric energy, overheat electrical devices, generate vibration and interference, and then affect the aging and service life of the lines. In order to effectively reduce the harmonic problems caused by different levels of the power system, it is necessary to analyze the harmonic components. In this paper, the BP neural network learning algorithm is introduced into the harmonic problems of the power system. The mapping relationship between input and output signals is obtained by using the BP neural network algorithm, and the harmonic frequency, amplitude, and phase contained in the obtained data are analyzed. According to the type of equipment with problems in the operation of the power system and the rapid diagnosis of existing defects, the problems are quickly located and the causes are analyzed. The practical results show that the BP neural network learning algorithm proposed in this paper has higher detection accuracy and analysis speed for the difficult problems in the power system.

## 1. Introduction

When harmonic issues of the power system are studied, massive data on the operation of equipment are accumulated, which can reflect the historical problems of the equipment and the related solutions [1, 2]. Historically, no effective data analysis has been conducted, and the relevant data are often stored in the corresponding system. Moreover, the equipment issues in the power system are resolved through maintenance, personnel's specialized expertise, and pragmatic experience accumulated over time because the equipment in the power system has functional deficiencies and the operation is complicated. In the case where historical issues are resolved by the BP neural network-based learning algorithm and the results of the case study are kept in the relevant platform, a database for maintenance cases of the power system equipment can be established. It will facilitate maintenance personnel in various areas for query, learning, and reference in real time to improve their communication so that they can share experience with each other and perform troubleshooting efficiently [3, 4].

As a reference, historical cases can help new maintenance personnel master the process of equipment operation and maintenance in the power system and improve their competency rapidly, which is vital for the effective diagnosis of the equipment later. According to the abovementioned analysis, combined with the data mining algorithm and bidirectional networks in the long- and short-terms, and random conditions, the research on the power system harmonic issue is completed to address the problems in the power system harmonic process effectively [5, 6]. By constructing the power system equipment knowledge graph of the ontology model, power system equipment failure is identified by the BP neural network-based learning algorithm. Accurate detection of the system frequency is the basis for better realizing harmonic detection and suppression. At the same time, it is also the key core problem of applying active filtering. The quality of detection directly determines whether the active filter can achieve harmonic compensation well. Hence, accurate real-time acquisition of harmonic data is required. When fundamental components can be measured accurately and quickly from the distorted waveform, the detection and suppression of higher harmonics can be accomplished. Sedzro et al. proposed a stochastic model of risk perception. This stochastic method considers the uncertainty of energy production and market price to maximize revenue and minimize loss risk. Chen et al. proposed a power management mechanism to meet the delay constraints of broadcast applications and the scheduling of scan aware packets, so as to provide a better quality of service for applications with multiple rates. Zhang et al. proposed an intelligent detection and the diagnosis system, which can reliably detect dangerous operating conditions online. The best trade-off between detection and diagnosis accuracy and detection and diagnosis is achieved. Muntean et al. proposed a solution for monitoring indoor and outdoor environmental parameters, including low-cost, easy to deploy wireless power devices, and cloud applications for managing, storing, and visually recording data. There are also some researches on harmonic detection and diagnosis of the power system. With the rapid development of artificial intelligence technology, the artificial neural network algorithm is gradually introduced into the harmonic analysis process of the power system, which is mainly divided into an adaptive linear neural network and the BP neural network learning algorithm. Both of these two algorithms can quickly detect the harmonic components, but they also have their own drawbacks. The adaptive linear neural network needs to clearly obtain the conditions for accurate harmonic analysis at the fundamental frequency; the window and the interpolation FFT algorithm can be used to detect the harmonic frequency, and the adaptive linear neural network algorithm can achieve better results in detecting the harmonic interpolation and phase process. The BP neural network algorithm can be used for harmonic detection; because there is uncertainty in the data training process, usually it needs to be trained for a long time before use, or there may be untrainable and local minima. Data acquisition is performed according to the convergence situation, so it cannot be applied to actual scenarios; however, the BP neural network learning algorithm has high accuracy and flexibility in real-time harmonic detection, and there is no strict limit on the number of samples collected. In addition, the BP neural network learning algorithm has the advantages of fast learning speed, no local minimum value, and consistent approximation performance for any nonlinear function, which can be applied to the harmonic detection of the power system.

Under the synchronous sampling of power system harmonics, the BP neural network algorithm will not produce spectral omission. According to this characteristic, it can be analyzed that by adjusting the sampling interval of the sampling sequence again, the harmonic signal of asynchronous sampling can be converted into a quasisynchronous signal. Relying on the BP neural network-based learning algorithm, this paper conducts technical analysis and harmonic research for the difficult problems in the power system, so as to reduce or eliminate the synchronization error.

## 2. Basic Correlation Algorithms

Assuming that the neural network has m layers with *N*_*i*_, *N*_*I*_, and *Nm* neurons in the input *I* in each m layers, respectively. In the BP neural network algorithm, *Xp* is variable inputs; Op is practical variable outputs [7, 8]; *Tp* is expected outputs. *ωi*/*jk* is the weight of the neuron *j* in the *i*-th layer on neuron *k* in the *i* + 1 layer; *Oi*/*j* is internal scalar outputs of neuron *j* in the *i*-th layer; *θi*/*j* is the threshold of neuron *j* in the *i*-th layer; *ui*/*j* is all inputs of neuron *j* in the *i*-th layer; *f* is the activation function. The variables have relationships as follows:

(1) $$\begin{array}{c} u_{j}^{i}=\sum_{k=1}^{N_{i-1}}\omega_{jk}^{i-1}o_{k}^{i-1},\\ o_{j}^{i}=f\left(u_{j}^{i}\right)=\frac{1}{1+\exp\left[-\left(u_{j}^{i}-\theta_{j}^{i}\right)\right]}. \end{array}$$

Input of neuron *j* in the hidden layer:

(2) $$\begin{array}{c} u_{j}=\sum_{i}\omega_{ij}o_{i}. \end{array}$$

Output of neuron *j* in the hidden layer:

(3) $$\begin{array}{c} o_{j}=f\left(u_{j}\right). \end{array}$$

Input of neuron *k* in the output layer:

(4) $$\begin{array}{c} u_{k}=\sum_{j}\omega_{jk}o_{j}. \end{array}$$

Output in the output layer:

(5) $$\begin{array}{c} o_{k}=f\left(u_{k}\right). \end{array}$$

The error function *E* of the neural network can be expressed as follows:

(6) $$\begin{array}{c} E=\frac{1}{2}\sum_{k}{\left(t_{k}-o_{k}\right)}^{2}. \end{array}$$

Weight adjustment is performed on the network in the gradient descent direction of *E* by the gradient descent method [9, 10], and calculation is conducted according to the equation as the following:

(7) $$\begin{array}{c} \Delta W_{jk}^{i}=-\eta \frac{\partial E}{\partial \omega_{jk}^{i}}=-\eta \left(\frac{\partial E}{\partial u_{jk}^{i+1}}\right)\frac{\partial u_{jk}^{i+1}}{\partial \omega_{jk}^{i}}=-\eta \delta_{k}^{i}\frac{\partial u_{jk}^{i+1}}{\partial \omega_{jk}^{i}}. \end{array}$$

where *η* is the learning efficiency coefficient, that is, the step size.

(8) $$\begin{array}{c} \delta_{k}^{i}=-\frac{\partial E}{\partial u_{k}^{i+1}}=-\frac{\partial E}{\partial o_{k}^{i+1}}\frac{\partial o_{k}^{i+1}}{\partial u_{k}^{i+1}}\\ \frac{\partial u_{k}^{i+1}}{\partial \omega_{jk}^{i}}=\frac{\partial \left(\sum_{k=1}^{Ni}\omega_{hk}^{i}o_{h}^{i}\right)}{\partial \omega_{jk}^{i}}\\ f\left(u_{k}^{i+1}\right)=\frac{1}{1+\exp\left(-u_{k}^{i+1}\right)}\\ \frac{\partial o_{k}^{i+1}}{\partial u_{k}^{i+1}}=f\left(u_{k}^{i+1}\right)=\frac{\exp\left(-u_{k}^{i+1}\right)}{{\left(1+\exp\left(-u_{k}^{i+1}\right)\right)}^{2}}=f\left(u_{k}^{i+1}\right)\left(1-f\left(u_{k}^{i+1}\right)\right)=o_{k}^{i+1}\left(1-o_{k}^{i+1}\right). \end{array}$$

In the hidden layer, node *Oi*+1/*k* is as follows:

(9) $$\begin{array}{c} \frac{\partial E}{\partial o_{k}^{i+1}}=\sum_{h=1}^{N_{i+2}}\frac{\partial E}{\partial u_{h}^{i+2}}\frac{\partial u_{h}^{i+2}}{\partial o_{k}^{i+1}}=-\sum_{h=1}^{N_{i+2}}\partial_{h}^{i+1}\omega_{kh}^{i+1}\\ u_{j}^{i}=\sum_{k=1}^{N_{i-1}}o_{k}^{i-1}\omega_{kj}^{i-1}\\ \delta_{k}^{i}=o_{k}^{i+1}\left(1-o_{k}^{i+1}\right)\sum_{h=1}^{N_{i+2}}\delta_{k}^{i+2}\omega_{kh}^{i+2}. \end{array}$$

When *Oi*+1/*k* is the node of the output layer:

(10) $$\begin{array}{c} \frac{\partial E}{\partial o_{k}^{i+1}}=t_{k}-o_{k}\\ \delta_{k}^{i}=-\frac{\partial E}{\partial u_{k}^{i+1}}=-\frac{\partial E}{\partial o_{k}^{i+2}}-\frac{\partial o_{k}^{i+1}}{\partial u_{k}^{i+1}}=\left(t_{k}-o_{k}^{m}\right)o_{k}^{m}\left(1-o_{k}^{m}\right). \end{array}$$

When the *i* + 1 layer is used as the output layer:

(11) $$\begin{array}{c} \Delta W_{jk}^{i}=\eta \left(t_{k}-o_{k}^{m}\right)o_{k}\left(1-o_{k}\right)o_{j}^{i}\\ \delta_{k}^{i}=\eta \left(t_{k}-o_{k}\right)o_{k}\left(1-o_{k}\right)\\ \Delta \theta_{k}^{i}=-\frac{\partial E}{\partial \theta_{k}^{i}}\left(t_{k}-o_{k}\right)o_{k}\left(1-o_{k}\right). \end{array}$$

The following can be obtained if the *i* + 1 layer is hidden:

(12) $$\begin{array}{c} \Delta W_{jk}^{i}=\eta o_{k}^{i+1}\left(1-o_{k}^{i+1}\right)\left(\sum_{h=1}^{N_{i+2}}\delta_{h}^{i+1}\omega_{kh}^{i+1}\right)\\ \delta_{k}^{i}=o_{k}^{i+1}\left(1-o_{k}^{i+1}\right)\left(\sum_{h=1}^{N_{i+2}}\delta_{h}^{i+1}\omega_{kh}^{i+1}\right)\\ \Delta \theta_{k}^{i}=-\eta \frac{\partial E}{\partial \theta_{k}^{i}}o_{k}^{i+1}\left(1-o_{k}\right)\left(\sum_{h=1}^{N_{i+2}}\delta_{h}^{i+1}\omega_{kh}^{i+1}\right). \end{array}$$

## 3. Harmonic Analysis with BP the Neural Network-Based Learning Algorithm

The characteristics of data are indicated using the proposed BP neural network algorithm for the power system with harmonic “drawbacks” as the target of analysis [11, 12]. For the purpose of mining and applying harmonics data of the power system, this paper builds a power system harmonics research platform, which mainly includes three layers (data, ontology, and application). In the data layer, harmonic data are processed by the BP neural network-based learning algorithm according to power equipment based on the historical records of harmonic issues, which has provided a basis to analyze the power system harmonic problem effectively. The ontology layer in the system is mainly to build the relationship between objects based on the algorithm, and then, the harmonic problem in the power system is formed. In the business layer, the data obtained are shared via the ontology layer. The BP neural network learning algorithm for power systems is a model extensively applied in the analysis of harmonic issues. In the study of harmonic problems in the power system, text features and CRF can be extracted by leveraging the advantages of the bidirectional storage network in the long term to accomplish the mission of sequence labeling and analyze harmonic issues.

Assuming that the optimized power data conversion range does not exceed the constraints, it can be generated in a random way and compared before and after the combination of harmonic signal operation and optimization to ensure multiobjective data.

If the optimized target exceeds the boundary range, the random generation method is used for modification. For a single-point objective of neuronal harmonic signals before and after optimization of harmonic signal manipulation, in order to ensure that the optimization target can transform the data, it is necessary to select any optimization target *h*_*r*_ as this conversion factor and leave it to the subsequent target. For other conversion targets, a random number *R* can be generated arbitrarily within the range of 0 to 1, and meanwhile, whether a multitarget crossover operation is required is determined according to the random number and the harmonic signal probability modification.

(13) $$\begin{array}{c} u_{h,n,g+1}=\left\{\begin{array}{cc} v_{h,n,g+1}, & R\leq P\;or\;h=h_{r}\\ x_{h,n,g}, & R>p, \end{array}\right.. \end{array}$$

where *u*_*h*,*n*,*g*+1_ in equation (13) is the *h*-th objective of the (*g* + 1)-th generation obtained after the harmonic signal operation; *v*_*h*,*n*,*g*+1_ is the (*g* + 1)-th generation neuron after the multiobjective optimization target, *x*_*h*,*n*,*g*_ is the *h*-th target of the *g*-th generation neuron before completing the harmonic signal, and *p* is the probability value of the harmonic signal.

Different fitness functions are selected based on different operating modes, and the optimal neuron is used to maintain the multiobjective differential evolution algorithm calculation. In this article, a binary coding method is used to indicate whether a component is faulty or not with a data bit. The collective size is 40. Natural selection refers to the operation of selecting superior neurons and eliminating inferior neurons from the collective [13, 14]. This paper adopts the competition method. The harmonic signal adopts the point harmonic signal method with a certain probability P, that is, a harmonic signal point is randomly selected in the neuron column, and the two neurons are partially exchanged before and after this point. Generation of new neuron by combining selection and harmonic signals, some permanent loss of information caused by selection, and harmonic signals can be avoided. Local random search can be performed by the multiobjective differential evolution algorithm to ensure its effectiveness. Meanwhile, the multiobjective differential evolution algorithm maintains the diversity of the group, and the optimization operation is also a measure to prevent the algorithm from premature. Based on the traditional multiobjective gap evolution algorithm, the following improvements are made. In terms of forming the initial neuron (giving an initial value), the neuron where the component failure occurs is formed like the component-related protection fault, and the neuron which generates the component failure and neurons without component failure are formed.

The symmetrical sigmoid function can be mathematically expressed as follows:

(14) $$\begin{array}{c} f\left(u\right)=\frac{1}{1+e^{-\lambda u}}. \end{array}$$

Thus, the asymmetric function for sigmoid is as follows:

(15) $$\begin{array}{c} f\left(u\right)=\frac{1-e^{-\lambda u}}{1+e^{-\lambda u}}. \end{array}$$

The internal *λ* is used as the function gain, which determines the function slope in the nonsaturated range; a larger *λ* indicates a steeper curve. From the characteristics of the S-function curve, it can be concluded that when it is used as the excitation function, since the middle is the high-gain region, it can adapt to weaker signals; and because the two ends are in the low-gain region, it can adapt to weaker signals and enhance the generalization of the neural network.

The principle of *δ* learning rule is as follows: assuming that the weight of the neuron is adjusted to minimize the function *F*(*w*). If the current weight of neuron is *w* (*t*), then the weight at the next moment is as follows:

(16) $$\begin{array}{c} w\left(t+1\right)=w\left(t\right)+\Delta w\left(t\right) \end{array}$$

In the formula, Δ*w*(*t*) is the weight adjustment direction at the current time point, and it is expected that each adjustment satisfies the following formula:

(17) $$\begin{array}{c} F\left(w\left(t+1\right)\right)<F\left(w\left(t\right)\right)\sqrt{a^{2}+b^{2}}. \end{array}$$

Conduct Taylor series expansion on *F*(*w*(*t* + 1)) to get the following formula:

(18) $$\begin{array}{c} F\left(w\left(t+1\right)\right)=F\left(w\left(t\right)+\Delta w\left(t\right)\right)\approx F\left(w\left(t\right)\right)+g^{T}\left(t\right)\Delta w\left(t\right). \end{array}$$

In formula (18), *gT*(*t*) = Δ*F*(*w*(*t*)) | *w* = *w*(*t*) is the gradient vector of F(*w*) at *w*(t).

(19) $$\begin{array}{c} \Delta w\left(t\right)=-cg\left(t\right). \end{array}$$

In the formula, *c* is the learning rate, which generally takes the smallest positive number, that is, a smaller value in the negative gradient direction is taken as the weight correction amount. Thus, the last term of equation (18) on the right side must be a negative value; then, the formula (18) will be automatically met according to the basic principle of the gradient method.

If any signal *f*(*t*) with period *T* is Fourier-expanded, the following can be obtained:

(20) $$\begin{array}{c} f\left(t\right)=a_{0}+\sum_{n=1}^{\infty }c_{n}\cos\left(n\omega t+\phi_{n}\right), \end{array}$$

where *ω* is the angular velocity value of the signal at the fundamental frequency. When *n* = 1, it corresponds to the parameter of the fundamental signal. Its magnitude and phase are expressed as follows:

(21) $$\begin{array}{c} \left\{\begin{array}{c} c_{1}=\sqrt{a_{1}^{2}+b_{1}^{2}},\\ \phi_{1}=tg^{-1}\left(-b_{1}/a_{1}\right), \end{array}\right.\\ \left\{\begin{array}{c} a_{1}=\frac{2}{T}\int_{t_{0}}^{t_{0}+T}f\left(t\right)\cos\;\omega t\;dt,\\ b_{1}=\frac{2}{T}\int_{t_{0}}^{t_{0}+T}f\left(t\right)sin\omega t\;dt. \end{array}\right.. \end{array}$$

The actual Fourier coefficients represent the content of cos*ω*t and sin*ω*t in the detected signal *f*(*t*). Therefore, if a certain signal is assumed, the corresponding fundamental wave component can always be obtained, that is, the signal waveform of the system and the fundamental wave component are always in a one-to-one correspondence. If the space formed by the full signal is set to be *f*(*A*), and the corresponding space formed by the fundamental wave components is *f*(*B*), it is proved that the mapping from *f*(*A*) to *f*(*B*) is an injective relation.

As a forward neural network that uses error to learn backwards, massive studies have been conducted on the BP neural network, and nonlinear mapping capacity is one of its essential functions. It is divided into input layer, hidden layer, and output layer. The three layers are mostly fully interconnected, but there is no interconnection relationship between units in the same layer. When a network is provided for a learning sample, the activation value of neurons propagates from the input layer through each intermediate layer to the output layer. After the neurons in each layer of the output layer obtain the input response of the network, they will reduce the error between the target output and the actual output. From the output layer to the middle layer, the connection weights are modified layer by layer, and finally back to the input layer. Only when the hidden layer has sufficient neurons, nonlinear mapping of input and output can be completed in 3-layer networks.  Figure 1 shows the structure of the BP neural network.

Here, the input of the network is the measurement target signal, xi is one of the *m* sample values, and yj is the fundamental wave component at the corresponding moment (*i* = 1, 2, 3,…, *n*, and *j* = 1, 2, 3,…, *n*).

(1) In its structure, neuron counts in each layer (input, output, and hidden) are designed, respectively [15]
  (a) Determine the neuron count in the input layer. The set of sample data with a certain pattern should include various types of patterns as much as possible, and the distribution of the samples should also meet the distribution in its practical application as much as possible. Assuming that the Fourier decomposition expansion of the nonsinusoidal periodic signal in the power system is shown in equation (21), the sampling period is 32 points per cycle, that is, fs = 1600 Hz, so there are 32 neurons in the input layer.
    (22) $$\begin{array}{c} f\left(t\right)=a_{0}+\sum_{n=1}^{\infty }c_{n}\cos\left(n\omega t+\varphi_{n}\right). \end{array}$$
  (b) The number of output layer units is determined to be 32, corresponding to the instantaneous value of the fundamental wave at the corresponding sampling time
  (c) In accordance with the number of layers and the famous Kolmogorov theorem, when there are sufficient nodes in the hidden layer, a neural network with a hidden layer can approach nonlinear function at any accuracy, so the fundamental wave detection network in this paper adopts the hidden layer.
  (d) Determination of hidden layers and neurons therein. In practice, hidden layer neurons can be selected empirically or by trial-and-error methods. According to the empirical formula, the neuron count in the hidden layer is as follows:
    (23) $$\begin{array}{c} s=\sqrt{0.43mn+0.12n^{2}+2.54m+0.77n+0.35}+0.15. \end{array}$$
  There are 98 nodes in the hidden layer. *m* is the neuron count in the input layer, *s* is the neuron count in the hidden layer, and *n* is the neuron count in the input layer.
  (e) Activation function selection: in this paper, an asymmetric S-function is selected for the activation function, and all input parameters and output parameters are normalized for samples. In this paper, the asymmetric sigmoid function is selected, and its standard input and output range is [0, 1].
  (f) The selection of the initial weight and the initial value of the weight must satisfy that the state of the superposition of the input of each neuron's approach to zero. Ensure that in the initial training state, all neurons are in the more sensitive area of the activation function, and try to avoid appearing in the insensitive area of the function. Since the activation function used in this paper is an asymmetric S function, the initial weight selected in this section is a set of random values between [0, 1]
  (g) Determination of the expected error: after the trend of training the network is on the right track, slowly reduce the error to 10–5, and train the network again. According to the abovementioned analysis, this paper designs a BP neural network including three layers: input, hidden, output, with 32, 98, and 32 neurons, respectively.
(2) Formation of training samples

Samples are critical for neural network learning. The information contained can directly affect the performance of the network. Whether the sample set is representative determines the learning effect of the network; the sample set size is used to describe a training set (data quantity and data distribution). As shown in Figure 2, a sample set of a pattern should contain as many types of patterns as possible, and the actual distribution of the samples should meet the actual application situation as much as possible. Since the system contains many nonlinear loads, most of the distortion waveforms generated are odd-ordered, but the proportion of harmonics is not very large; a higher harmonic order generally indicates a smaller amplitude. The signal of the system voltage or current may also contain a DC component, that is, when its average value is not equal to zero.

Therefore, the sample set selected from current/voltage signals of the grid in this paper is the following combination:

1. Fundamental wave, DC component, and harmonic components (3, 5, 7)
2. Fundamental wave and harmonic components (3)
3. Fundamental wave and harmonic components (5)
4. Fundamental wave and harmonic components (7)
5. Fundamental wave and harmonic components (3, 5)
6. Fundamental wave and harmonic components (3, 7)
7. Fundamental wave and harmonic components (5, 7)
8. Fundamental wave and DC components
9. Only fundamental components

The proportion of the DC component is about 0.1 times that of the fundamental wave; the amplitude of the 3rd harmonic component (Figure 3) is no larger than 0.3 times; the amplitude of the 5th harmonic is smaller than 0.2 times; the amplitude of the 7th harmonic is smaller than 0.025 times.

The specific training sample set is *X* = [*X*_1_, *X*_2_, *X*_3_, *X*_4_, *X*_5_, *X*_6_, *X*_7_, *X*_8_, *X*_9_], *X*_1_,…, *X*_9_ are respectively as follows.

(24) $$\begin{array}{c} X_{1}=0.1+\sin\left(\omega t\right)+0.3\;\sin\left(3\omega t\right)+0.2\;\sin\left(5\omega t+\frac{\pi }{4}\right)+0.025\;\sin\left(7\omega t+\frac{\pi }{3}\right),\\ X_{2}=\sin\left(\omega t\right)+0.3\;\sin\left(3\omega t\right)\\ X_{3}=\sin\left(\omega t\right)+0.2\;\sin\left(5\omega t+\frac{\pi }{4}\right)\\ X_{4}=\sin\left(\omega t\right)+0.025\;\sin\left(7\omega t+\frac{\pi }{3}\right)\\ X_{5}=\sin\left(\omega t\right)+0.3\;\sin\left(3\omega t\right)+0.2\;\sin\left(5\omega t+\frac{\pi }{4}\right)\\ X_{6}=\sin\left(\omega t\right)+0.3\;\sin\left(3\omega t\right)+0.025\;\sin\left(7\omega t+\frac{\pi }{3}\right)\\ X_{7}=\sin\left(\omega t\right)+0.2\;\sin\left(5\omega t+\frac{\pi }{4}\right)+0.025\;\sin\left(7\omega t+\frac{\pi }{3}\right)\\ X_{8}=0.15+\sin\left(\omega t\right)\\ X_{9}=\sin\left(\omega t\right). \end{array}$$

where *ω* = 2*π*f, and the value range of *f* is [49.5, 50.5].

## 4. Simulation Example

For the purpose of ensuring that erroneous information in the harmonic signal of the power system can be detected by the BP neural network algorithm, the harmonic signal information data obtained in this experiment is used. At this time, the harmonic problem of the power system will be parameterized according to the actual situation, as shown in Table 1, where *λ* is the regularization coefficient of *L*2; optimizer is the optimizer of the algorithm solution (Adam is the estimation algorithm of the adaptive moment, SGD is the descent algorithm of the stochastic gradient); *N*_Hidden_dim_ is the neuron count in the BiLSTM hidden layer; *N*_Epoch_ is the rounds of sample training; *N*_Batch_size_ is the sample size of each batch selected; *γ*_Learning_rate_ is the algorithm learning rate; *N*_Embedding_dim_ is the vector distribution dimension when harmonics are converted to vectors; *γ*_Dropout_ is the random dropping rate of neurons.

The performance of the model is assessed based on three indices: precision (*P*), recovery (*R*), and *F*1 according to equations (2)–(4). The results in 4 control groups are shown in Table 1.

It can be observed from the abovementioned simulation results that the neural network and Prony algorithm can be used to analyze the harmonics of the power system. In the absence of noise, the width value and phase have high precision, plus white noise with only 0.001 times the fundamental wave. However, due to the large width of the fundamental wave, even if a small white noise is added, the measurement accuracy of harmonics is greatly reduced.

Comparing the power system harmonic problem proposed in this paper (control group 1), Table 2 shows three indices (accuracy, recovery, and F1) in the experimental group based on CRF, BiLSTM-softmax, and Seq2Seq-attention, respectively, under the natural language generation model. Table 2 indicates that the proposed power system harmonic method has better accuracy (87.12%), recovery (86.46%), and F1 (0.8679) than CRF, BiLSTM-softmax, and Seq2Seq-attention, respectively. Furthermore, an accuracy of above 90% can be achieved when three entities of the fault solution for location in the Q&A dataset of power service are identified and extracted by CRF. The test accuracy of the dataset used in this paper is only 70.01%, which also verifies the advantages of the study of harmonic problems in power systems.

In order to further verify the effectiveness of the BP neural network algorithm, this paper selects the sample data of harmonics when different angle deviations as the test data and conducts analysis and simulation verification of the algorithm. This paper collects and analyzes harmonic samples according to the changes of the specific rectification angle, specifically, which can be divided into five angles of *α* = 0°, *α* = 30°, *α* = 60°, *α* = 90°, and *α* = 120° for network diagnosis. In order to further detect the harmonic diagnosis results of the network, the corresponding training samples are used for analysis, and the actual output of the neural network is represented by 0 and 1 to facilitate comparison with the expected output.

The output of the neural network is reasonably processed using the judgment principle, and the processed data can correctly reflect the diagnosis results of the harmonic wave.  Figure 4 shows the harmonic diagnosis accuracy when *α* is taken as 0°, 30°, 60°, 90°, and 120° respectively.

It can be seen from the results in Figure 4 that the BP neural network algorithm has good classification performance and high efficiency of intelligent detection and diagnosis.

## 5. Conclusion

In the normal running power system, speed changes in the synchronous generator will lead to the change of the frequency of the power system, which is in line with the basic principle of the harmonic current detection method. On the basis of analyzing the shortcomings of independent detection methods, a BP neural network-based learning algorithm is proposed from the essential function of the active power filter to the improve power quality and reduce total harmonic distortion rate to analyze the reason of frequency fluctuation of the power system. The neural network is used to simulate the fundamental wave signal to obtain the required fundamental wave frequency; the harmonic parameter estimation can achieve high accuracy. The research on the harmonic problem of the power system has been improved in the evaluation index, which can be used for providing a theoretical basis for plotting the knowledge graph, reading relevant data, conducting standardized processing, etc. in the power system. The harmonic issues in the power system can be effectively addressed based on the comparison of track records to ensure a more intelligent and suitable model for application scenes in practice. According to the test results, the proposed method can resolve the harmonic problems and detect the harmonic current in the power system using the active power filter at the harmonic detection stage.

## Figures and Tables

**Figure 1:** Structure diagram of the BP neural network.

**Figure 2:** Current linear neuron model.

**Figure 3:** Harmonic simulation model.

**Figure 4:** Harmonic diagnostic accuracy.

**Table 1:** Settings of model hyper-parameters.

Hyper-parameters	Value			
	Control group 1	Control group 2	Control group 3	Control group 4
*λ*	0.0001	0.001	0	0.0001
Optimizer	Adam	Adam	Adam	SGD
*N*_hidden_dim_	400	400	400	400
*N*_epoch_	40	40	40	40
*N*_batch_size_	35	35	35	35
*γ*_learning_rate_	0.001	0.001	0.001	0.001
*N*_embedding_dim_	200	200	200	200
*γ*_dropout_	0.4	0.4	0.4	0.4

**Table 2:** Comparison of model performance by experiments.

Models	Accuracy (%)	Recall (%)	*F*1
CRF	70.02	70.43	0.7142
BiLSTM-softmax	78.73	71.9	0.7714
Seq2Seq-attention	71.63	—	—
BP neural network learning	87.13	86.47	0.8779

## Data Availability

The data used to support the findings of this study are available from the corresponding author upon request.
